# Developments of Interfacial Measurement Using Cavity Scanning Microwave Microscopy

**DOI:** 10.1155/2022/1306000

**Published:** 2022-08-12

**Authors:** Zhenrong Zhang, Huanfei Wen, Liangjie Li, Tao Pei, Hao Guo, Zhonghao Li, Jun Tang, Jun Liu

**Affiliations:** ^1^Key Laboratory of Instrument Science and Dynamic Testing Ministry of Education, North University of China, Taiyuan 030051, China; ^2^Key Lab of Quantum Sensing and Precision Measurement, Shanxi Province, Taiyuan 030051, China; ^3^Institute of Instrument and Electronics, North University of China, Taiyuan 030051, China

## Abstract

In the field of materials research, scanning microwave microscopy imaging has already become a vital research tool due to its high sensitivity and nondestructive testing of samples. In this article, we review the main theoretical and fundamental components of microwave imaging, in addition to the wide range of applications of microwave imaging. Rather than the indirect determination of material properties by measuring dielectric constants and conductivity, microwave microscopy now permits the direct investigation of semiconductor devices, electromagnetic fields, and ferroelectric domains. This paper reviews recent advances in scanning microwave microscopy in the areas of resolution and operating frequency and presents a discussion of possible future industrial and academic applications.

## 1. Introduction

Over the past decade, one of the most significant advances in the field of microwave testing has been the emergence of scanning microwave microscopy [1–9]. There are two main types of scanning microwave microscope, categorized according to the source of the microwave signals at the scanning tip, with one type using a microwave resonator coupled to the tip of the probe using a small aperture and the other using a coaxial transmission line directly attached the tip of the atomic force microscopy (AFM) cantilever. Regardless of whether the small aperture of the probe is contained in a sharp tip or a cavity, the formation of the microwave image is accomplished through the capture of the microwave reflectance either in magnitude or in phase, as well as by the simultaneous probe scanning across the specimen surface [10–13]. In this review, we focus on the resonant cavity-type scanning microwave microscope.

The scanning microwave microscope can be used to study the electromagnetic properties of a sample via an interaction with a nanoscale scanning probe. Scanning microwave microscopy allows quantitative measurements of dielectric constants and losses in materials. The use of this approach enables simultaneous high-speed, noncontact, and nondestructive measurements to be made [14–16]. In some cases, the microwaves can penetrate into the sample, providing opportunities for tomographic analysis [17]. Due to these advantages, scanning microwave microscopy can achieve nanoscale near-field measurements, something of great use in future applications of high-resolution microwave image generation.

In this review, we present recent advances in the research of scanning microwave microscopy. The current progress in applications and development of the technique are reviewed here, including its limitations and advantages, as well as the scope for further developments. The paper begins with a discussion of the basic design and subsequent improvements in instrumentation for scanning microwave microscopy. Then current applications of the technique are discussed. Finally, conclusions and a discussion of possible future developments are made.

## 2. Basic Design and Improvements in Instrumentation for Scanning Microwave Microscopy

The use of microwaves permits the generation of decaying or evanescent electromagnetic fields at discontinuities in waveguides and the use of these highly-confined fields for microscopy [18]. This type of microscopy is sometimes referred to as “scanning microwave impedance microscopy” (SMIM), “near-field scanning microwave microscopy” (NSMM), or “near-field microwave microscopy” (NFMM), but here, we will uniformly refer to the technique as “scanning microwave microscopy” (SMM). There are many kinds of signal analysis used to construct the images, such as the change in the Quality (*Q*) factor of the resonant cavity, the change in capacitance between the probe and the sample, the frequency drift, and the *S*_11_ and *S*_21_ values of the microwave signal. In recent years, most experimental systems have used vector network analyzers to acquire the required signals, although some researchers continue to build their own signal acquisition systems. Materials with different properties cause different obstacles to microwave conduction related to the composition, structure, purity, defect, and impurity content of the samples. This allows microwave microscopy to use changes in the conduction of the microwaves in the near-field as a diagnostic test. Using microwaves as a test signal has the advantages that optical and acoustic signals lack, such as strong penetration, no damage to the sample, and short relaxation time.

Current approaches to scanning microwave microscopy follow similar lines. The signal resonates through the resonator, and the field is concentrated by the use of a tip much smaller than the wavelength of the microwaves, resulting in a strong local measurement of the sample [19]. Local storage of part of the signal is noted in the near-zone and evanescent waves. The rest of the signal is partially absorbed by the specimen, partially reflected to the transmission line, and partially dispersed in the form of far-field illumination. The specimen response can be captured by monitoring the height- and position-dependent variations of the reflected or dispersed signals [20]. The reflected microwave signal decays quickly and can be solved analytically using transmission line theory [21–25].  Figure 1 shows the key components of a typical near-field microwave microscope [23].

The microscope consists of a microwave source, a coaxial resonator coupled to the microwave generator (through a decoupling capacitor or inductor), a detector to measure the reflected signal from the resonator, and a frequency-following circuit (FFC) [26]. The instrument shown in Figure 1 uses a half-wavelength resonant cavity, but many scanning microwave microscopes use a four-wavelength resonant cavity, as shown in Figure 2 [20].

This approach uses a significantly faster technology called phase-sensitive detection. By adjusting the phase shifter, the difference in phase between the resonator and a reference signal is made 90° in the absence of the sample under the tip. The amplification, fusion, and subsequent feedback of this signal to the VCO (voltage-controlled oscillator) are made possible by the proportionality of the phase detector output to the magnitude of the phase shift, thereby achieving the oscillator phase locking at *f*_*r*_. For quantification of the *f*_*r*_ shift and *Q* under this approach, a diode detector is utilized to separately determine the amplitude of the resonator output signal and the error signal of the phase lock loop. By moving the specimen under the resonator-tip assembly, the acquisition of images is possible while documenting the variations in *f*_*r*_ and *Q*.

A series lumped equivalent resonant circuit in series (Figure 3) can be used to model the SMM system. The angular resonant frequency can be calculated from $\omega_{r}=2\pi f_{r}=1/\sqrt{\text{LC}}$, where *L* and *C* are the effective inductance and capacitance, respectively, and *f*_*r*_ is the resonant frequency [20, 25]. The impedance of the lumped elements can be used to quantify the sample-tip interaction *Z*_*t*_ = *R*_*t*_ + **i***X*_*t*_, with *Z*_*t*_ being a function of the geometry of tip, the distance of the tip from the sample, and the electrodynamic properties of the sample. A detailed theoretical analysis between the tip of the needle and the sample is given in reference [23].

## 3. Early Developments in Scanning Microwave Microscopy

Scanning microwave microscopy is a useful tool for studying the surface and internal structure of materials. It is used to test a variety of physical quantities, including dielectric and ferroelectric dielectrics and the properties of materials such as semiconductors, metals, superconductors, and biological specimens. However, there are still challenges remaining to its wide-scale adoption, the most significant of which is the existence of a large common-mode signal arising in part from noise. Reducing the noise signal is an area of intense current study to permit the broadening of applications for the technique through higher resolution and clearer images.

Thanawalla et al. [25] proposed a tip-structured probe employing a high-quality resonator and a novel shielding structure to shield the probe tip from far-field components. This permitted the imaging of the dielectric constant and loss tangent of dielectric materials at the spatial resolution of 100 nm and sensitivity of *δε*/*ε* ≈ 1 × 10^−5^. The quantitative complex electrical impedance microscopy is also possible using model analysis. As microwave wavelengths in metals are four orders of magnitude smaller than those in free space, they did not study metals with their system.

Williams et al. [26] achieved a resolution of 25 nm with their system. They utilized a resonant circuit to provide a method for detecting capacitance changes between the tip and a surface below 100 *μ*m with a sensitivity of 1 × 10^–19^ F at a bandwidth of 1 kHz. The feedback control circuit was used, and the tip was scanned at a fixed distance from the sample to provide a noncontact method of surface profiling. They presented images of both conducting and nonconducting structures, demonstrating a sensitivity limit for capacitance imaging of below 10 nm, and showing capacitance imaging at the 25 nm scale (Figure 4).

Manassen et al. [27] demonstrated atomic-resolution imaging using a hybrid scanning tunneling/near-field microwave microscope. The microwave channels of the microscope conform to the resonant frequency and quality factor of a coaxial microwave resonator, which is built into the STM scan head and coupled to the probe tip.  Figure 5 shows some of the images that they obtained. They found that they could obtain atomic-resolution images by adopting the microwave channel of the *μ*-wave STM provided that the tip sampling distance was within the tunneling state [19]. They conjectured that the atomic contrast in the microwave channels was caused by a GHz frequency current flowing through the tip-sample tunnel junction. They imaged both HOPG and Au(111) surfaces. GHz atomic-resolution images allow material properties such as those arising from elemental selectivity/sensitivity phenomena to be observed, including dielectric relaxation and electron spin resonance [27]. In addition, the MHz bandwidth of the resonators used in this research proved suitable for use in high-speed spectroscopic measurements at the atomic scale.

Biani et al. [28] described the imaging of graphene sheets using a homebuilt double-channel scanning probe microscope that performed both near-field broadband scanning microwave microscopy and STM. They incorporated conversion in the time-domain to generate microwave images of superior quality with nanometric resolution. For the time-domain elucidation of the desired signal, an inverse Fourier transform was implemented. They deposited the graphene specimens on a SiO_2_ substrate and overlaid them with gold. The results appeared to demonstrate a drastic variation in impedance in the vicinity of the flake edges, which probably suggests a build-up of charge.

Jooyoung et al. [29] conceived an SMM system that comprised a coaxial *λ*/4 resonator with a tunable cavity that was coupled to a sharp probe tip. When the operational frequency *f* ranged between 1 and 1.5 GHz, they were able to achieve better spatial resolution and sensitivity compared to that of the near-field image (4 *μ*m) of a YBa_2_Cu_3_O_y_ film that was deposited on a MgO substrate [29]. By appropriately tuning the length of the resonance cavity, the probe could be made even more sensitive. The spatial resolution and sensitivity variations with the length of the cavity were adjusted using the resonance cavity tuning. This system has the potential to extend the measurement range by extending the frequency range and lowering the operating temperature.

Bertness et al. [30] demonstrated that SMM is suitable for use in determining the photoresponse of photovoltaic materials whose lateral resolution may be of submicrometer scale. In this approach, an RF-STM (radiofrequency scanning tunneling microscopy) tip is coupled to a microwave cavity, whose resonance frequency is around 4.5 GHz. The load on the cavity is altered by the additional mobile carriers near the tip of the probe. Quantification of these alterations is accomplished by measuring the shifts in the *Q* factor and resonance frequency. In the case of the GaAs and Cu (ln, Ga) Sez solar cell material, the conductivity variation determination under blue light irradiation was easily achievable. As modeling of this behavior improves, this approach should become sensitive enough to quantify the sample conductivity fluctuations on both the absolute and relative scales. The use of SMM for the testing of photovoltaic materials is a very fruitful area of future application, as photovoltaic materials are of increasing importance in the modern world.

Talanov et al. [31] designed a microwave probe for near-field scanning with a sampling diameter of around 10 *μ*m. This is the smallest sample volume yet attained in near-field microwave microscopy and constrains > 99% of the gross sampling reactive energy for the probe so that the response is almost irrelevant to the properties of samples outside this zone. The probe comprises a balanced stripline micrometer-sized resonator (4 GHz) that can carry out noncontact, nondestructive testing. Its applicability to the spatially localized metrology of electrical quantities is especially high.

Tabib-Azar et al. [32] investigated several issues concerning the development of evanescent microwave probes (EMP) and discussed the applicability of such probes in materials research. They determined that these probes were superior in terms of spatial resolution to those with lower dielectric constants and superior in terms of spatial resolution to those with lower permittivity. In the case of magnetic dipole probes, they found that their resolution was not identically reliant on the dielectric constant of the substrate. They attributed this lack of appreciable dependence to the prevailing reliance of the magnetic field curves on the radius of the probe wire loops and the irrelevance of the loop dimension to the permittivity of the substrate. In semiconductors, the use of EMP enabled imaging of the conductivity fluctuation, as well as the recombination lifetime. Their use also allowed the acquisition of the nonuniform behavior of composites, metals, insulators, balsa wood, and a plant leaf. The EMP promises broad applicability in investigating botanical and biological materials, as it achieves the nondestructive and noncontact imaging of these materials via appropriate media like air.

In summary, since the earliest days following its inception, scanning microwave microscopy has found a very wide range of applications in testing material dielectric constants, morphology, optoelectronic materials, biological samples, and so on. Moreover, its increase in resolution, coupled with its nondestructive nature, provided a good research basis for the subsequent development of SMM.

## 4. Recent Developments in Scanning Microwave Microscopy

In this section, we summarize the recent advances in the use of scanning microwave microscopy to study material properties, morphology, chip imaging, and biological testing, respectively.

### 4.1. Recent Advances in the Use of SMM to Determine Material Properties

Bakli et al. [11] reported the use of an interferometric procedure in place of classic resonant approaches, which utilized repeated passive devices with superior stability and accuracy. Their fading probe, which has high impedance, is compatible with current metrological measurement systems, and the method has the advantages of being broadband and having high measurement precision and convenience of operation. Using this integration of interferometry and near-field microscopy, they could obtain high measurement sensitivity without using large and expensive resonators. They also developed a new calibration model for relating the near-field reflectance measurement to the local properties of the test sample.

Fecioru-Morariu et al. [33] reported a method for acquiring the distribution diagram of high-frequency conductivity for an oxide-coated ferromagnetic membrane as thin as 200 nm based on the SMM-derived *Q*. Circuit analog estimation was used to assess the electrical properties for the resonator. The interaction between the sample and tip was modeled using FEA so that the resonant frequency and *Q* values corresponding to the sample were retrievable [34]. The simulation was verified using a specimen of thin Cu membrane to quantify the simulated *Q* variation with the conductivity plot. They then explored how the nonmagnetic application of Al_2_O_3_ on AF (antiferromagnetic) IrMn films affected the high-frequency conductivity of the films by calculations that provide high-frequency conductivity values for these thin-film samples.

Imtiaz et al. [35] tested the widely used quasistatic deem bedding procedure for characterizing bulk materials with SMM tips. To properly characterize conducting materials, the extra loss mechanism resulting from the antenna impedance fluctuation into the near-field that was above the plane of the conducting ground must be considered [36–38]. This loss is determined by the material conductivity, and the loss is considerable in the case of materials considerably exceeding 10^3^ S/m [35]. Quasistatic models were found to be acceptable for fused silica and silicon, as the variation of impedance attributable to the plane boundary proximity with materials was ignorable when the conductivities were below 10^3^ S/m. They also introduced an SMM-based strategy for material differentiation via complex permittivity magnitude by plotting the variation of the product (Δ*f*/*f*_0_)(*Q*/*Q*_0_) with the tip height.

### 4.2. Testing the Topography of the Material

Zhang et al. [8] reported a method that could correct the skewing and denoising of SMM images, significantly enhancing the spatial resolution of the images, as can be seen in Figure 6. Through electromagnetic simulation, they obtained the optimal approach to increasing the electric field strength at the tip of the needle. This includes reducing the length of the tip protruding from the coaxial cavity, the distance between the tip and the sample, and the diameter of the tip. They scanned a Cu film grid and compared the half-height widths of the test curves with and without tip optimization to obtain a method for enhancing the sensitivity of the SMM system. The detection sensitivity was greatest when the tip protruded 3 mm from the cavity, the distance between the tip and the sample was 1.44 *μ*m, and the diameter of the tip was 1.6 *μ*m. In addition to the Cu thin-film grid, they also tested *f*_*r*_, *S*_11_, and *Q* images of coin textures, lithographic masks, and leaf veins, and the test images became sharper than the originally obtained blurred images using their tilt correction method.

Bagdad et al. [39] designed and fabricated a scanning microwave microscope for characterizing semiconductor structures, as shown in Figure 7. Their SMM system utilizes a homemade coaxial cavity resonator that uses a network analyzer as the signal source. The inner resonator conductor is linked to a sharpened tungsten tip made, which was electrochemically prepared. Semiconductor structural metrics, including the resonance frequency *f*_*r*_, the quality factor *Q*, the reflection coefficient *S*_11_, and the transmission *S*_21_ for the resonant cavity, were scanned with the sharpened tip of the probe while maintaining the tip-sample distance within the near-field zone. Due to the interaction of the probe tip with the test sample, the metric parameters undergo fluctuations, showing correlations with the dielectric properties and topography of the tiny material zone beneath the probe tip. This makes it possible to generate a 2D image of the *f*_*r*_, *Q*, *S*_11_, and *S*_21_ parametric progression on the surface of the test sample.

Gao and Xiang [40] used an SMM instrument for measuring the interconnect and interline capacitance in a noncontact mode at the femtofarad level with the aid of a miniature tester device [40]. Their procedure is applicable to the investigation of the variation in electrical parameters in integrated circuit interconnects while generating parameters for subsequent statistical design. They also explored its applicability to the determination of low-dielectric losses and interconnect line resistance. The geometry of their tester device may be suitable for the microwave elucidation of diverse functional nanomaterials, including carbon nanotubes, nanofibers, nanowires, and nanoribbons through the connection of the test object between the 2 interconnect lines.

Gregory et al. [41] utilized a wire probe with a globular tip of a diameter of approximately 0.1 mm as a modification of the cavity perturbation type. Given the enrichment of the field at the zone closest to the specimen, the measurement resolution using this probe is on the order of microns, which is considerably less than the diameter of the tip, particularly at a high dielectric constant. They presented both an innovative SMM design and a novel calibration algorithm, as well as a novel calibration reference (polar liquids). They used Laplace “complex frequencies” for the first time in the computational and calibration outcomes, which permitted the accurate measurement of losses in highly lossy materials. In addition, for a microwave microscope having a line probe, a beam deflector was designed.

### 4.3. Imaging of the Subsurface of the Sample

The microwave signal can penetrate certain media to a depth sufficient to obtain subsurface information of the sample. Pearanda-Foix [42] described the use of scanning microwave microscopy techniques to identify security markings on banknotes. Their system included a stand-alone vector network analyzer to allow the reflection response of a near-field coaxial probe to be measured. They combined displacement laser and cavity perturbation techniques to investigate the correlation between the dielectric properties of the sample and the resonant response of the probe. The system was able to measure subsurface subfabricated images, as shown in Figure 8.

### 4.4. Imaging of the Local Electric Field Properties of Nanomaterials

Measurements of the local density of states and local surface resistance can reveal how changes in the local density of states because of impurities, defects, grains, carrier bias, etc., affect local resistance on the nanometer scale [43, 44].

Tadashi et al. [45] measured the local density of states and the local surface resistance in low local surface resistance materials through the local measurements of tunneling spectra and sheet resistance within the boundary region of the gold deposition and nondeposition zones on the HOPG by SMM. Their results showed significant differences in the local resistance around the boundary as well as differences in the tunneling spectra. They combined their system with STM to measure the local density of states as well as local surface resistance on the nanoscale. Their work demonstrated that this approach is a useful tool to study the effect of local disorder on electrodynamics and measure the local properties of nanomaterials.

### 4.5. Imaging of the Local Magnetic Properties of Metal Samples

Magnetic materials are essential materials in modern science and technology [46, 47]. The sensitivity of SMM to magnetic properties makes it suitable for use in testing magnetic materials. Lee et al. [48] demonstrated the sensitivity of their homemade SMM system to magnetism. They used a loop probe that differed from the usual probe and were able to observe an obvious contrast between ferromagnetic and paramagnetic materials that was both qualitative and quantitative. Their results are shown in Figure 9, where the maximum change in the FMR field is about 230 Oe in both images. As can be seen, a large amount of image smearing occurs near the edges of the sample.

### 4.6. Imaging the Radiated Power of Microwave Chips

In recent years, diagnosing problems within highly integrated microwave chips has received a lot of attention. The use of SMM to test chips offers opportunities for noncontact testing and a small scanning zone.

Lin et al. [49] have reported a resolution enhancement method for subsurface noninvasive application of imaging based on an SMM system that comprises an EMP (evanescent microwave probe), a VNA (vector network analyzer), a data capture system, and a motorized *XYZ* stage with high resolution. Thanks to the interferometric-based broadband matching architecture, adjustment of the sample–probe electromagnetic coupling is achievable so that the measurement can be highly sensitive at arbitrary frequencies between 2 and 18 GHz. The image processing approach uses the PSD (position/signal difference) and ARS (adaptive robust statistical) methods. Valid error rectification is possible with the proposed solution because of the measurement noise and specimen tilt so that the quality of imaging can be upgraded for the noninvasive assessment.

Kleismit et al. [50] tested a homemade *λ*/4 evanescent microwave sensor. The sensor can be used for elucidating the local electromagnetic properties of materials, as illustrated in Figure 10. The resonator intrinsic inherent spatial resolution of the resonator has been corroborated through experimental demonstration. The first-order approximation estimation of the sensitivity related to the sample–probe tip-sample interaction was presented for conductors, dielectrics, and superconductors. An estimation of the intrinsic sensitivity inherent to the resonant probe was also presented. The sensitivity of the probe is in the range of micrometers. The system is also capable of generating the local complex permittivity values for dielectric, conductor, and superconductor sample specimens, which is achieved through the determination of the resonant frequency shift of the resonant coaxial probe toward the surface of the sample as the tip moves toward the sample surface. The resonant frequency shift is measured relative to the reference resonant frequency, which is the resonance frequency when the tip is 1 *μ*m from the surface.

### 4.7. Imaging of Dynamic Microwave Fields

The use of SMM offers a means of imaging the microwave field distribution when the chip is working in real-time. Guo et al. [51, 52] used a scanning microwave microscope with a microwave resonant cavity with a *Q* of 209 to identify nano defects on the waveguide surface in chips. They obtained microwave waveguide microwave field signals with a resolution of up to 1 pW and plotted the microwave field distribution in microwave core operation with a resolution that can reach 15 nm, as shown in Figures 11 and 12. This method offers high resolution and the capability for online monitoring for microwave chip evaluation and screening and, as such, could have far-reaching applications in chip fabrication, chip inspection, and nanostructure detection.

Chen et al. [52] proposed a simple method for testing very weak microwaves using a homemade scanning microwave microscope detection system consisting of a *λ*/4 tunable resonant cavity and a tungsten tip. They solved the technical problem of impedance matching and inhibited the background noise by enhancing the number of cycles of the coupling loop. Using this approach, the efficiency of electromagnetic wave loading into the tip sampling system is improved, and the measured values of thermal parameters of the chip are obtained using a noncontact scanning mode.

### 4.8. Imaging of Samples in Extreme Environments

The demand for nondestructive testing in high-temperature environments has been increasing. Online or in-service high-temperature NDT systems will save time and energy, lower costs, and enhance efficiency [53].

Reznik and Yurasova [53] demonstrated the use of a homemade quartz lamp radiation module as a heater coupled to a homemade microwave microscope probe. They tested the amplitude and phase of a hexagonal honeycomb lattice at room temperature and 50°C at a resonant frequency of 1 GHz. Their work confirmed that multibands could be used for subsurface detection and superresolution imaging at high temperatures. Their system could clearly distinguish metal gratings with line and gap widths of 0.5 mm at 1 GHz, and the resolution reached *λ*/600 (Figure 13).

### 4.9. Imaging of Biological Samples

The attractiveness of microwave technology for biological applications stems from a combination of its sensitivity to water and dielectric contrasts and its noncontact and nondestructive nature [54].

Wu et al. [55] used a homemade scanning microwave microscope that allowed contact/tapping mode imaging of both nonconductive and conductive specimens [55]. Their system used a flexible CNT (carbon nanotube tip) carbon nanotube tip, which facilitated the upgrade in image quality and also protected the specimen surface from scratches. By manipulating the SMM and CNT tip in tapping mode, they depicted the *f*_*r*_ and *S*_11_ amplitudes in a designated scan region and acquired photoresist stripes, gold-patterned numbers, and clear B_4_G_12_ (corneal endothelial) cell images (Figure 14). In the acquired images, the cytoplasm and nucleus are distinguishable from the remaining part of the cell and peripheral medium, suggesting the possible SMM application in cellular imaging. This work lays the foundation for the further development and application of SMM techniques for soft matter imaging in biosciences. In Figures 14(c) and 14(d), the red area represents the nucleus, the yellow and green areas represent the outline of the cell, and the dark blue area corresponds to the cytoplasm, showing the quality of the image.

Farina et al. [56] presented a primitive interferometric procedure-based NFMM instrument for dielectric elucidation in liquid media, where a vector network analyzer was integrated with an interferometric-based matching architecture and a novel fast microstrip probe that was prepared via a silicon deposition technique. This approach allowed a more-sensitive determination of microwave signals at the desired frequencies from 1 to 26 GHz. The system also had the virtue of simplicity.

Haddadi et al. [16] used SMM and scanning capacitance microscopy (SCM) to assess the presence of fullerene (*C*_60_) in dry cancer cell membranes after appropriate exposure. They analyzed the SMM data in the time and frequency domains. This preliminary study suggests that both SMM and SCM can be adopted to indicate the presence of *C*_60_ in cells, as shown in Figure 15. Fullerene is a nanoparticle being actively explored for possible uses in biology and medicine because of its lipophilic nature and ability to dope or permeate cell membranes.

Zhang et al. [8] reported a method that can correct the skewing and denoising of SMM images, significantly improving the spatial resolution of the images. They detected and obtained parametric images of *f*_*r*_, *S*_11_, and *Q* of the veins of leaves, as illustrated in Figure 16. After the application of the tilt correction, the images were much clearer than the original blurred images.

## 5. Conclusions and Future Prospects

Scanning microwave microscopy has developed into a very broad research topic since its introduction and is favored by many researchers due to the nondestructive advantages of microwave testing [57–59]. It has now been successfully applied to characterize surface and subsurface samples at the nanoscale spatial resolution, exploring properties such as dielectric constant, doping concentration, and resistivity. In terms of the investigation of the electrical properties of materials, scanning microwave microscopy shows advantages over other conventional microscopies, being unaffected by temperature changes, the presence or absence of a vacuum, and can even work in strong magnetic field environments. It also has good prospects for the online detection of chip electromagnetic fields in real-time. However, there is still room for research in terms of microwave signal resolution and image optimization methods, and this is likely to prove a target for future exploration. At the same time, methods for transmitting microwaves more conducive to the tip radiation method are also being explored, such as the use of special AFM probes made of platinum [60] and micro- and nanoprocessing on silicon nitride cantilevers [61–63]. To improve the accuracy and sensitivity of microwave signal detection, we still need to both reduce the size of the probe under limited process conditions and reduce the influence of the noise signal on the test signal. We anticipate that the application scope of scanning microwave microscopy will continue to expand.

## Figures and Tables

**Figure 1:** Schematic diagram of the key components of a half-wavelength cavity-type near-field scanning microwave microscope.

**Figure 2:** Schematic diagram of the key components of a *λ*/4  cavity-type near-field scanning microwave microscope.

**Figure 3:** Equivalent circuit of a cavity-type near-field scanning microwave microscope.

**Figure 4:** Grayscale and line scan capacitance images of an array of 50 nm diameter holes, 50 nm apart. The structure is an l00 nm-thick PMMA film that is overcoated with 20 nm of gold. The field of view of a 370 nm square [26].

**Figure 5:** A 300 × 300 nm^2^ area of Au(111), showing the atomic-resolution microwave signal images of *f*_*r*_ using a hybrid STM/SMM system. The STM bias line and the current preamplifier are disconnected from the setup during SMM imaging [27].

**Figure 6:** An enhanced grid contour image and *f*_*r*_ parameter image of a copper film after tilt correction [8].

**Figure 7:** The 2D distribution of the resonant frequency (GHz) on a 50 *μ*m-width gold layer deposited on top of a SiO_2_/Si substrate [39].

**Figure 8:** Images of the watermark included in a 20 EUR banknote obscured by a metallic mask [42].

**Figure 9:** Images of an LSMO single-crystal taken at 6.037 GHz at a sample–probe separation of 10 *μ*m. (a) ∆*f* image of the LSMO sample at an external field *H*_ext_ = 1317 Oe, chosen to give a minimum unloaded *Q* factor at the center of the sample, and (b) unloaded *Q* factor image at an external field *H*_ext_ = 1411 Oe, chosen to give a minimum ∆*f* at the center of the sample. A background frequency shift has been subtracted from (a). The dashed line presents the approximate location of the sample [48].

**Figure 10:** Application of the ARS method to case 3 (10 *μ*m-80 *μ*m) [49]. (a) Before the ARS processing. (b) After the ARS processing.

**Figure 11:** Spatial plots of the section of the bare copper wire and coplanar waveguide. (a) MW field distribution of the bare copper wire section and (b) MW field distribution of the CPW section [51].

**Figure 12:** Spatial plots of the MW waveguide in the MW chip. (a) MW chip, (b) MW waveguide in the MW chip, (c) surface of the MW waveguide, (d) MW field simulation of the MW waveguide, (e) two-dimensional image of the MW field distribution in the MW waveguide, (f) the corresponding three-dimensional image of the MW field distribution in the MW waveguide, and (g) MW power in the two MW waveguides [51].

**Figure 13:** (a) Images of the scanning amplitude and phase of the inner honeycomb core at 20°C and 50°C, (b) the linear distribution of the phase, and (c) the phase image after edge detection processing [53].

**Figure 14:** (a) The optical image of corneal endothelial cells (B_4_G_12_) on a glass coverslip, (b) the phase contrast image of a pair of adjacent B_4_G_12_ cells, (c) the resonant frequency *f*_*r*_ 3D plot, (d) *S*_11_ amplitude 3D plot, (e) resonant frequency *f*_*r*_ contour plot, and (*f*) *S*_11_ amplitude contour plot [55].

**Figure 15:** (a) Time-domain SMM image of MCF-7 cells treated with fullerene and (b) the simultaneous STM image (processed to remove the tilt plane). The taller cells are 3 *μ*m [16].

**Figure 16:** SMM image correction in the imaging of leaf veins. (a) *f*_*r*_ and (b) *Q* image of original data. (c) Tilt-corrected *f*_*r*_ image and (d) *Q* image [8].
